This article has been retracted.

# Berberine Improves Kidney Function in Diabetic Mice via AMPK Activation

**DOI:** 10.1371/journal.pone.0113398

**Published:** 2014-11-19

**Authors:** Long Zhao, Li-Na Sun, Hui-Bin Nie, Xue-Ling Wang, Guang-Ju Guan

**Affiliations:** Nephrology Research Institute, the Second Hospital of Shandong University, Jinan, Shandong, China; University of Hull, United Kingdom

## Abstract

Diabetic nephropathy is a major cause of morbidity and mortality in diabetic patients. Effective therapies to prevent the development of this disease are required. Berberine (BBR) has several preventive effects on diabetes and its complications. However, the molecular mechanism of BBR on kidney function in diabetes is not well defined. Here, we reported that activation of AMP-activated protein kinase (AMPK) is required for BBR-induced improvement of kidney function in vivo. AMPK phosphorylation and activity, productions of reactive oxygen species (ROS), kidney function including serum blood urea nitrogen (BUN), creatinine clearance (Ccr), and urinary protein excretion, morphology of glomerulus were determined in vitro or in vivo. Exposure of cultured human glomerulus mesangial cells (HGMCs) to BBR time- or dose-dependently activates AMPK by increasing the thr172 phosphorylation and its activities. Inhibition of LKB1 by siRNA or mutant abolished BBR-induced AMPK activation. Incubation of cells with high glucose (HG, 30 mM) markedly induced the oxidative stress of HGMCs, which were abolished by 5-aminoimidazole-4-carboxamide ribonucleoside, AMPK gene overexpression or BBR. Importantly, the effects induced by BBR were bypassed by AMPK siRNA transfection in HG-treated HGMCs. In animal studies, streptozotocin-induced hyperglycemia dramatically promoted glomerulosclerosis and impaired kidney function by increasing serum BUN, urinary protein excretion, and decreasing Ccr, as well as increased oxidative stress. Administration of BBR remarkably improved kidney function in wildtype mice but not in AMPKα2-deficient mice. We conclude that AMPK activation is required for BBR to improve kidney function in diabetic mice.

## Introduction

Diabetes mellitus represents a global threat for premature morbidity and mortality [1]. Diabetic nephropathy (DN) is a major chronic microvascular complication of diabetes and characterized by a progressive increase in albuminuria and a decline in glomerular filtration rate [2]. Mechanisms underlying nephropathy in diabetes include a range of hemodynamic and metabolic factors [3]. A growing number of studies support that the generation of reactive oxygen species (ROS) as a common downstream pathway of most of these mechanisms ultimately leads to inflammation and fibrosis [4]. However, the exact pathogenesis of DN is complex and poorly understood.

Berberine (BBR) is an isoquinolone alkaloid found in plants such as *Phellodendron chinense* and *Coptis chinensis*. In traditional Chinese medicine, BBR from *Coptidis rhizoma* is used as a constituent of the herbal medicine Huanglian [5]. In this form it is reported to exert anti-fungal, anti-bacterial/viral, and anti-oncogenic effects, as well as a beneficial effect on diabetes, and anti-atherogenic properties [6], [7]. Several mechanisms are reported to be associated with the beneficial properties of BBR including improvement of sugar and lipid metabolism [8]. BBR has also been reported to reduce the incidence of diabetes through suppression of oxidative stress. Whether BBR exerts its beneficial effects in DN and the molecular targets are undefined.

The AMP-activated protein kinase (AMPK) is a heterotrimeric protein composed of α, β, and γ subunits. The α subunit imparts catalytic activity, while the β subunit contains a glycogen-binding domain that also regulates the activity and the γ subunit forms the broad base of the protein and is required for AMP binding. AMPK is well-conserved among eukaryotic cells and is expressed in endothelial cells of different origins. Activation of AMPK requires phosphorylation of Thr172 in the activation loop of the α subunit and is mediated by at least two kinases, Peutz-Jeghers syndrome kinase LKB1 (LKB1) and Ca^2+^/calmodulin-dependent protein kinase kinase. AMPK has been shown to mediate angiogenic and anti-inflammatory effects [9]. Indeed, BBR has been reported to activate AMPK in several cell types, such as endothelial cells, smooth muscle cells [10], cardiomyocytes [11], [12], cancer cells [13], β-cell [14], liver cells [15], macrophages [16], [17], adipocytes [18]. Based on these reports, we hypothesized that the protective effects of BBR on kidney function in diabetes may be due, in part, to the ability of BBR to stimulate AMPK to suppress oxidative stress.

## Materials and Methods

### Materials

BBR, streptozotocin (STZ) and 5-aminoimidazole-4-carboxamide ribonucleoside (AICAR) were purchased from Sigma (St. Louis, MO, USA). BBR was dissolved in DMSO to make a 500 mM stock solution (0.1% v/v final concentration) and stored at −80°C. AMPKα1/2 siRNA, LKB1 siRNA, and all primary antibodies were purchased from Cell Signaling Company or Santa Cruz Biotechnology. The siRNA delivery agent Lipofectamine 2000 was purchased from Invitrogen (Carlsbad, CA). Other chemicals were obtained from Sigma-Aldrich (St Louis, MO) unless otherwise indicated.

### Animals

C57/BL6 wildtype (WT) mice (6–8 weeks of age, 20–25 g of bodyweight) were purchased from the animal department of Hunan Normal University. AMPKα2^-/-^ mice were generated by Viollet B [19]. They were maintained in a temperature-controlled (22°C) under a 12 h light/dark cycle, pathogen-free environment and fed a standard rodent chow diet and water ad libitum. Male WT mice, 8–12 weeks of age, 20–25 g, were obtained from the Jackson Laboratory (Bar Harbor, ME). A low-dose (50 mg/kg/day for 5 consecutive days) STZ induction regimen was used to induce pancreatic islet cell destruction and persistent hyperglycemia as described by the Animal Models of Diabetic Complications Consortium (http://www.amdcc.org). Hyperglycemia was defined as a random blood glucose level of >300 mg/dL for >2 weeks after injection. The animal protocol was reviewed and approved by the University of Shandong, Animal Care and Use Committee.

### Primary cell culture

For isolation of human glomerulus mesangial cells (HGMCs), collected kidney from surgery were washed twice with PBS at 4°C and cut into small pieces. These pieces were purified by 100-mesh sieve to get glomerular. Then the glomerular was incubated in a 0.2% collagenase solution at 37°C for 15–20 minutes. Cell pellets were incubated in 1640 medium with full components. Purity of HGMCs was confirmed through positive staining for collagen and fibronectin. The participants have provided their written informed consent. We recorded the general information and got the permission from the patients to use their kidneys for studying only. The study protocol was approved by the Ethical Committee of the Second Hospital of Shandong University.

### Adenovirus infections in cells

Ad-GFP, a replication-defective adenoviral vector expressing green fluorescence protein (GFP), served as control. An adenoviral vector expressing a constitutively active mutant of AMPK (AMPK-CA), was subcloned from a rat cDNA encoding residues 1-312 of AMPK and bearing a Thr172-to-Asp mutation (T172D) into a shuttle vector (pShuttle CMV [cytomegalovirus]). Cells were infected with GFP or AMPK-CA in medium with 2% feta calf serum overnight. The cells were then washed and incubated in fresh growth medium without feta calf serum for an additional 12 h before experimentation. Using these conditions, infection efficiency was typically >80%, as determined by GFP expression.

### Transfection of siRNA into cells

Transient transfection of siRNA was carried out according to Santa Cruz's protocol. Briefly, the siRNAs were dissolved in siRNA buffer (20 mM KCl; 6 mM HEPES, pH 7.5; 0.2 mM MgCl_2_) to prepare a 10 µM stock solution. Cells grown in 6-well plates were transfected with siRNA in transfection medium containing liposomal transfection reagent (Lipofectamine 2000, Invitrogen). For each transfection, 100 µl transfection medium containing 4 µl siRNA stock solution was gently mixed with 100 µl transfection medium containing 4 µl transfection reagent. After 30-min incubation at room temperature, siRNA-lipid complexes were added to the cells in 1.0 ml transfection medium, and cells were incubated with this mixture for 6 h at 37°C. The transfection medium was then replaced with normal medium, and cells were cultured for 48 h.

### Western blot analysis

As described previously [20], the protein content in total cell lysates or homogenized tissues was determined using the bicinchoninic acid protein assay reagent (Pierce, USA). Twenty micrograms of protein was separated by SDS-PAGE and then transferred to a membrane. The membrane was incubated with a 1∶1,000 dilution of primary antibody and a 1∶2,000 dilution of horseradish peroxidase-conjugated secondary antibody. Protein bands were visualized by enhanced chemiluminescence (GE Healthcare). The intensity (area × density) of the individual bands on western blots was measured by densitometry (model GS-700, Imaging Densitometer; Bio-Rad). The background was subtracted from the calculated area. The control was set to 100%.

### AMPK activity assay

AMPK activity was assayed using the SAMS peptide. The activity was determined in the presence and absence of AMP (200 µM). AMPK activity was calculated by determining the difference in activity between both conditions.

### Determination of kidney morphology

To assess the glomerular sclerotic injury, renal tissues were embedded in paraffin and 4 µm-thick sections were prepared for periodic acid schiff (PAS) staining. Glomerulosclerosis (GS) was evaluated by determining the percentage of glomeruli exhibiting sclerotic lesions (%GS). 200 consecutive glomeruli were examined for each mouse. The data were averaged. Lesion scores related to the glomerular and mesangial area were graded according to the following scale: 0 =  preservation of the architecture, 1 = 5-15% glomerular expansion or mesangial expansion and PAS positivity, 2 = 15–30% glomerular expansion or mesangial expansion and PAS positivity, 3 = 30–50% glomerular expansion or mesangial expansion and PAS positivity, and 4 = >50% glomerular expansion or mesangial expansion and PAS positivity, which was described previously [21].

### Renal function measurement

Blood samples were centrifuged at 2000 g for 10 min, serum were collected for measuring BUN by using a commercially available kit (ABIN, Cat: 577679). Urine samples were centrifuged in the same way to remove any suspended particles and the supernatant was used to detect 24-hour urine albumin protein by using Albumin Mouse ELISA Kit (abcam, Cat: 108792). The creatinine was measured with a Creatinine Companion kit (Exocell, Cat: 1012). The renal function was assessed by measurement of Cr clearance (Ccr) as urinary Cr X urine volume/serum Cr and expressed as milliliters per minute.

### Immunohistochemistry

The expressions of 3-nitrotyrosine (3-NT) and malondialdehyde (MDA) in kidney were measured by immunohistochemistry in paraffin embedded sections following the process as previously described [22]. All morphological analyses and cell counting were performed on blinded slides.

### Detection of ROS

Tissue or cell O_2_^-^ levels were measured using the DHE fluorescence/HPLC assay with minor modifications [23]. Briefly, tissues or cells were incubated with DHE (10 µM) for 30 min, homogenized, and subjected to methanol extraction. HPLC was performed using a C-18 column (mobile phase: gradient of acetonitrile and 0.1% trifluoroacetic acid) to separate and quantify oxyethidium (product of DHE and O_2_^-^) and ethidium (a product of DHE auto-oxidation). O_2_^-^ production was determined by conversion of DHE into oxyethidine.

### Statistical Analysis

Results are expressed as the mean ± SD. Statistical significance for comparison between two groups was calculated using the two-tailed Student's *t* test. To assess comparisons between multiple groups, analysis of variance (ANOVA) followed by the Bonferroni procedure was performed using the Graph-Pad Prism 4 program (GraphPad Software, Inc, San Diego, CA). A *P* value of <0.05 was considered to be statistically significant.

## Results

### BBR activates AMPK via Thr172 phosphorylation in time- and dose- dependent manner in cultured HGMCs

Earlier studies had established that phosphorylation of AMPK at Thr172 correlates with AMPK activity [24]. BBR is well characterized as a drug to protect diabetes and the vascular complications. To investigate whether BBR activates AMPK in kidney, confluent HGMCs was treated with varying concentrations of BBR from 10 to 200 µM in culture medium for 2 hours. AMPK activation was indirectly assessed by western blot analysis of AMPK phosphorylation at Thr172, which is essential for AMPK activity. As shown in Figure 1A, BBR of 100 µM did not affect phosphorylation of AMPK at 1 hour point. In contrast, BBR began to activate AMPK at 2 hours. Increasing incubating time of BBR (100 µM) further enhanced AMPK phosphorylation. In Figure 1B, the phosphorylation of AMPK gradually increased beginning from 25 µM after incubation with BBR for 2 hours and reached peak levels at 100 µM in HGMCs. BBR treatment did not alter total levels of AMPK (Figure 1A and 1B), suggesting that BBR-induced phosphorylation of AMPK was not due to altered expression of the total protein. In addition, increased AMPK phosphorylation was associated with elevated AMPK activity, as measured by the SAMS peptide assay [25] (Figure 1C).

**Figure 1:** BBR activates AMPK in cultured HGMCs. (**A**) Cultured primary HGMCs were incubated with BBR (100 µM) for indicated time after starvation overnight. AMPK thr172 phosphorylation in total cell lysate was detected by western blot. The blot is a representative of three blots from three independent experiments. *P<0.05 VS control. (**B**) Dose-dependent effects of BBR on AMPK-Thr172 phosphorylation in HGMECs. N is 3 in each group. *P<0.05 *VS* control. (**C**) Confluent HGMCs were treated with BBR (100 µM) for 2 hours. AMPK activity was assayed using the SAMS peptide as a substrate. N is 5 in each group. *P<0.05 VS control.

### BBR-induced AMPK phosphorylation in HGMCs is LKB1-dependent

To study how BBR activates AMPK, we suppressed LKB1 expression, which is an AMPK upstream kinase by applying siRNA in cells [26]. We found that LKB1 siRNA, but not control siRNA, inhibited BBR-induced phosphorylation of AMPK at Thr172 if LKB1 protein expression was silenced by siRNA (Figure 2A). These experiments offer solid support for the notion that LKB1 is required for BBR-induced AMPK activation in cells.

**Figure 2:** BBR-induced AMPK activation in cultured HGMCs is LKB1-dependent. (**A**) HGMCs were transfected with control siRNA or LKB1 siRNA for 48 h. Then cells were treated with BBR (100 µM) for 2 hours. AMPK thr172 phosphorylation in total cell lysate was detected by western blot. The blot is a representative of three blots from three independent experiments. *P<0.05 VS control. NS indicates no significance. (**B**) HGMCs were infected with adenovirus containing LKB1-WT, LKB1-S428A or LKB1-S307A for 48 h. The infected cells were then treated with BBR (100 µM) for 2 hours. AMPK-Thr172 phosphorylation was detected by Western blot. The blot is a representative blot from three independent experiments. *P<0.05 VS ad-GFP. NS indicates no significance.

We next evaluated whether LKB1 phosphorylation at Ser307 or Ser428 was required for BBR-induced AMPK activation [27]. Using site-directed mutagenesis, we developed an LKB1 mutant in which an amino acid essential for LKB1 activation, serine 307 or 428, was mutated to alanine. Since BBR treatment resulted in increased phosphorylation of AMPK in cells infected with adenovirus encoding WT-LKB1, we next investigated whether adenoviral overexpression of the LKB1 mutant would prevent BBR-induced phosphorylation of AMPK. As expected, LKB1-S307A or LKB1-S428A mutant did abolish BBR-enhanced phosphorylation of AMPK-Thr172 (Figure 2B). These data suggest that LKB1 is essential for BBR-induced AMPK activation in cells.

### Activation of AMPK attenuates HG-induced oxidative stress

Permanent hyperglycemia is the most common single cause of kidney failure. Oxidative stress and inflammation are proved to be critical for the pathogenesis of diabetes mellitus. In order to induce the injury of kidney cells, we mimicked hyperglycemia by using high glucose (30 mM D-glucose) in culture medium to treat HGMCs. As shown in Figure 3A and 3B, incubation of HGMCs with high glucose (HG) significantly increased the ROS productions. These results are consistent with previous report [25]. Further, activation of AMPK by AICAR (Figure 3A) or gene overexpression (Figure 3B) abolished HG-induced oxidative stress in HGMCs, indicating that HG-induced oxidative stress is AMPK-dependent.

**Figure 3:** AMPK upregulations by AICAR or gene overexpression attenuate HG-induced oxidative stress in cultured HGMCs. (**A**) HGMCs were incubated with D-glucose (30 mM) in presence or absence of AICAR (2 mM) for 12 hours. ROS productions were detected by DHE fluorescence. N is 5 in each group. ^*^ *P*<0.05 vs. control, ^#^ *P*<0.05 vs HG alone. (**B**) HGMCs infected with Ad-GFP or Ad-AMPK-CA for 48 hours were incubated with HG for 12 hours. ROS productions were detected by DHE fluorescence. The picture is a representative from 3 independent experiments. ^*^ *P*<0.05 vs. control GFP. NS indicates no significance.

### BBR via AMPK activation suppresses HG-induced oxidative stress

We next determined whether BBR suppressed HG-induced oxidative stress through AMPK activation. To test this notion, we performed siRNA transfection to knockdown AMPK α1 and α2 protein levels. As depicted in Figure 4A, the level of AMPK protein was silenced significantly by specific siRNA, but not control siRNA. As expected, BBR treatment dramatically suppressed HG-induced oxidative stress in cultured HGMCs as assayed by DHE fluorescence (Figure 4B and 4C). Collectively, these results demonstrate that AMPK plays a key role in BBR-reduced oxidative stress in HG-treated HGMCs.

**Figure 4:** BBR via AMPK activation reverses HG-induced oxidative stress in HGMCs. HGMCs were transfected with AMPKα1/2 siRNA for 48 hours. Then cells were pre-incubated with BBR (100 µM) for 30 minutes followed by treatment with D-glucose (30 mM) for 12 hours. (**A**) AMPKα protein expression in total cell lysates was assayed by Western blot. (**B**) ROS productions were detected by DHE fluorescence. (**C**) Quantitative data of ROS productions. N is 5 in each group. ^*^ *P*<0.05 vs. control, ^#^ *P*<0.05 vs HG plus control siRNA. NS indicates no significance.

### Hyperglycemia induces kidney dysfunction in STZ-injected mice

Then we investigated whether administration of BBR improved kidney function in diabetic mice. After 16-week STZ-induced hyperglycemia duration, morphology of kidneys from all mice was assayed by PAS staining (Figure 5A). Compared to control WT mice, hyperglycemia remarkably caused fibrosis, containing abnormal glomeruli. Similar to formation of glomerulosclerosis, diabetes also induced renal dysfunction as increased serum BUN (Figure 5B), decreased Ccr (Figure 5C), and enhanced urinary albumin excretion (Figure 5D).

**Figure 5:** BBR prevents hyperglycemia-induced renal dysfunction in *WT* but not in *AMPKα2^-/-^* mice. Permanent hyperglycemia in *WT* and *AMPKα2^-/-^* mice was induced by a low-dose STZ induction. All mice were received with or without BBR administration (200 mg/kg body weight daily) for 8 weeks after the stable diabetic model was established. At the end of experiments, mice were sacrificed. (**A**) Blood glucose in all mice. 5–10 mice in each group. ^*^ *P*<0.05 vs. WT alone, ^#^ *P*<0.05 vs STZ plus WT. NS indicates no significance. (**B**) Morphological and quantitative analysis of glomerulus by HE staining. a, WT; b, WT + STZ; c, WT + STZ + BBR; d, *AMPKα2^-/-^* + STZ; e, *AMPKα2^-/-^* + STZ + BBR. (**C**) Serum BUN, (**D**) creatine clearance rate (Ccr), and (**E**) urinary protein excretion were assayed. 5–10 mice in each group. ^*^ *P*<0.05 vs. control, ^#^ *P*<0.05 vs DM in WT. NS indicates no significance.

### Treatment of mice with BBR attenuates diabetes-induced kidney dysfunction in *WT* but not in *AMPKα2^-/-^* mice

Then we determined the effects of BBR on diabetes-induced renal dysfunction. Injection of STZ dramatically increased blood glucose in WT and *AMPKα2^-/-^* mice. Interestingly, the increases of blood glucose induced by STZ in *AMPKα2^-/-^* mice were slightly higher that WT mice. As shown in Figure 5B, BBR significantly inhibited the hyperglycemia-induced the formation of the glomerulosclerosis in WT but not in *AMPKα2^-/-^* diabetic mice. Quantitative analysis indicated that STZ significantly increased lesion score in WT mice. BBR remarkably reduced the lesion score in WT but not in *AMPKα2^-/-^* diabetic mice. Similarly, BBR reversed the increased serum BUN (Figure 5C), decreased Ccr (Figure 5D), and enhanced urinary albumin excretion (Figure 5E) induced by hyperglycemia, suggesting that AMPK is a key mediator to perform the protective effects of BBR in diabetic nephropathy.

### Diabetes-induced oxidative stress in kidney is reversed by BBR in *WT* but not in *AMPKα2^-/-^* mice

Pathophysiological processes of diabetes is extreme complex and controversial. A growing number of evidences showed that oxidative stress and inflammation might play important roles in the development of DN. We finally checked the oxidative stress in diabetic mice by assaying 3-NT and MDA, which are makers of peroxidation of protein or lipid [28]. As shown in Figure 6A, 6B, and 6C, our data showed that hyperglycemia increased the levels of 3-NT and MDA in kidney as compared to control group. Treatment of BBR significantly decreased levels of 3-NT and MDA in *WT* diabetic mice but not in *AMPKα2^-/-^* diabetic mice, suggesting BBR via AMPK activation reduced oxidative stress in diabetic mice.

**Figure 6:** BBR via AMPK prevents hyperglycemia-induced oxidative stress in mice. Permanent hyperglycemia in *WT* and *AMPKα2^-/-^* mice was induced by a low-dose STZ induction as described in method section. All mice were received with or without BBR administration (200 mg/kg body weight daily) for 8 weeks after the stable diabetic model was established. At the end of experiments, mice were sacrificed to detect MDA and 3-NT by IHC. (**A**) Representative pictures of MDA and 3-NT. (**B**) Quantitative analysis of 3-NT. (**C**) Quantitative analysis of MDA. 5–10 mice in each group. ^*^ *P*<0.05 vs. control, ^#^ *P*<0.05 vs DM in WT. NS indicates no significance.

## Discussion

In the present study, we have shown that LKB1-AMPK signaling mediates BBR-protected kidney function in diabetic mice. The underlying mechanism in this process is due to a novel pathway in which kidney dysfunction is inhibited by BBR as a result of AMPK activation. These findings indicate that AMPK pathway is an important mediator for kidney cell function and suggest that BBR therapy that modulates AMPK signaling may be beneficial in treating kidney dysfunction in diabetic nephropathy.

BBR is a natural compound isolated from plants and with multiple pharmacological activities [8]. The emerging role of BBR in modifying sugar and lipid metabolism has been verified in a large amount of experimental and clinical studies. Notably, due to the low toxicity, BBR could be used in diabetic patients with chronic hepatitis. Beneficial effects of BBR were also observed in combating diabetic complications [29]. Diabetes-related endothelial dysfunction, nephropathy, and neuropathy could be relieved after BBR administration. Recently, some groups reported that BBR has some protective effects in different stages of diabetes in rats, such as diabetic nephropathy [30]–[33]. However, this present study not only demonstrated that BBR improves kidney function and inhibits glomerular fibrosis in diabetic mice, but further uncovered the molecular mechanisms, which BBR activates LKB1-AMPK signaling to suppress oxidative stress in glomerulus mesangial cells. Most importantly, the protective effects of BBR on kidney function in diabetic mice were mediated by AMPK because BBR was unable to protect liver functions in *AMPKα2^-/-^* mice, indicating the important role of AMPK in BBR-induced beneficial effects. In fact, BBR has been reported to activate AMPK in vascular endothelial cells and suppressed formation of atherosclerosis [34], [35]. Combined with these observations, BBR would be explored to treat kidney and cardiovascular disease, which are related to diabetic complications.

Interestingly, we discovered that STZ-induced type 1 diabetes damaged renal function and induced glomerulosclerosis in mice. This is inconsistent with Qi's report [36]. We reasoned that the discrepancy should be due to the time difference of persistent hyperglycemia. Actually, Zhang M et al. also reported that the kidney function and the morphology of glomerular started to be abnormal at the 6^th^ week and were serve at the 9^th^ week during hyperglycemia [37], as well as the 8^th^ week which we reported. Another issue is that the relationship between AMPK and ROS remains controversial. Recently, Kumar Sharma et al. demonstrated that superoxide is increased by AMPK, which is renal-protective [38]. In fact, AMPK functions as a redox sensor and modulator, in which slight increase of ROS can activate AMPK. However, activation of AMPK reduces ROS production. The disagreement would be due to the different level of ROS productions. Further studies are required to test these possibilities.

In summary, we have demonstrated that BBR attenuates diabetic nephropathy *in vivo* via AMPK activation. In addition, the improvement of kidney function by BBR appears to be mediated by suppression of oxidative stress. The data presented here support the concept that AMPK may be an important therapeutic target for treating diabetic nephropathy and other kidney diseases related to oxidative stress. Therefore, till now, there is no report about the effects of BBR on diabetic nephropathy in clinical patients, indicating the potential application for BBR on treating diabetic kidney disease in patients in future.
